# Pediatric Glaucoma: A Literature's Review and Analysis of Surgical Results

**DOI:** 10.1155/2015/393670

**Published:** 2015-09-16

**Authors:** Gianluca Scuderi, Daniela Iacovello, Federica Pranno, Pasquale Plateroti, Luca Scuderi

**Affiliations:** NESMOS Department, Faculty of Medicine and Psychology, Sapienza University, Via grottarossa 1035-1039, 00139 Rome, Italy

## Abstract

The purpose of this paper is to review the surgical options available for the management of pediatric glaucoma, to evaluate their advantages and disadvantages together with their long-term efficacy, all with the intent to give guidelines to physicians on which elements are to be considered when taking a surgical decision. Currently there is a range of surgical procedures that are being used for the management of pediatric glaucoma. Within these, some are completely new approaches, while others are improvements of the more traditional procedures. Throughout this vast range of surgical options, angle surgery remains the first choice in mild cases and both goniotomy and trabeculotomy have good success rates. Trabeculectomy with or without mitomycin C (MMC) is preferred in refractory cases, in aphakic eyes, and in older children. GDIs have a good success rate in aphakic eyes. Nonpenetrating deep sclerectomy is still rarely used; nevertheless the results of ongoing studies are encouraging. The different clinical situations should always be weighed against the risks associated with the procedures for the individual patients. Glaucomatous progression can occur many years after its stabilization and at any time during the follow-up period; for this reason life-long assessment is necessary.

## 1. Introduction

Pediatric glaucoma is a condition characterized by an elevated intraocular pressure (IOP) and optic nerve damage and it can be potential cause of blindness [1].

The most common classification is the following.

1. Primary congenital glaucoma, including isolated idiopathic developmental anomalies of the angle structures.
2. Glaucoma arises in a series of systemic diseases some associated with iridocorneal trabeculodysgenesis syndrome such as Axenfeld Rieger syndrome or Peter's anomaly [2], the phakomatoses in particular Sturge-Weber syndrome and its variants [3–5]. It can be associated also with neurofibroamatosis [6, 7], homocystinuria, Lowe's syndrome, mucopolysaccharidosis, juvenile xanthogranuloma [8, 9].
3. Secondary glaucoma associated with acquired ocular disease.

Depending on the timing of the diagnosis and on features and circumstances of presentation of the glaucoma, aspects that must all be very carefully evaluated, surgery represents the mainstay of treatment, while topical medication may be needed for additional IOP control following surgery or as a temporary measure.

Currently, there are different surgical options, including newer surgical procedures that are improvements of the traditional ones; these in association with the use of antimetabolites and of new viewer systems contribute greatly to the improvement of the prognosis of this disease.

The purpose of this paper is to analyze the surgical options available for the management of pediatric glaucoma and to evaluate their advantages and disadvantages together with their long-term efficacy, all with the intent to give guidelines to physicians on which elements are to be considered when taking a surgical decision.

## 2. Angle Surgery: Goniotomy and Trabeculotomy

### 2.1. Goniotomy

The initial approach for primary congenital glaucoma is still angle surgery: goniotomy in the case of a clear cornea or trabeculotomy in the case of a cloudier cornea (Tables 1 and 2). Experienced surgeons have a high rate of success with this technique. Nonetheless, the patient should fit within certain criteria such as the primary congenital glaucoma with no other ocular or systemic anomalies, first diagnosed at least one month after birth but before on year of age, and the corneal diameters need to be less than 14 mm.

Goniotomy was described for the first time by Barkan in 1948 [10] although his pioneer was actually de Vincentis who first performed it in 1893 [11]. The main aims and steps of this procedure have remained the same throughout the years; however, some modifications have been introduced, such as the use of a surgical microscope, the introduction of new goniolens (Koeppe, Barkan, Ritch), and the use of viscoelastic material to protect the cornea and lens.

The surgical steps include entering the anterior chamber, using a goniotomy knife to perform a corneal incision so as to reach the opposite side of the chamber and then incise the trabecular meshwork for 100–110 degrees, visualized using a goniolens. One of the most recently introduced is the Ritch lens; this is a direct lens that allows a 160 degree view of the angle and obstructs only half of the cornea thus making it easier to introduce the goniotomy instrument into the eye while the goniolens is in place. In case of failure it can be repeated.

Barkan in 1953 described the result of his 17 years of work with goniotomy in congenital glaucoma; he reported an 80% success rate in 188 eyes, with postoperative IOP values less than 20 mmHg without medications [12].

In 1982 Shaffer described results in 287 operated eyes. Glaucoma was considered cured if the intraocular pressure remained below 20 mmHg without medication for at least six months and cupping of the optic nerve was either the same or improved. The success rate was 76.7%. However, when the signs or symptoms of glaucoma were present at the birth or above the age of 24 months, the success rate was close to 30%. In contrast the success rate improved to 94% in cases diagnosed between the age of 1 and 24 months after one or two goniotomies [13]. This difference can be explained by the microstructural changes that are detectable in the different age groups; indeed patients over the age of 24 months are known to have less cellularity and more collagenous tissue with respect to younger patients. In the same work he also described that after 15 years of follow-up 3 patients had an increase between 20 and 30 in IOP and therefore required medical therapy [13].

Another study discussed long-term goniotomy complications; in particular the authors described a risk of relapse of glaucoma for at least 15 years. Patients whose symptoms of congenital glaucoma presented at birth were more likely to relapse than those whose symptoms developed in the first few months of life. Furthermore, eyes that required multiple goniotomies in infancy were more likely to relapse than those controlled by a single procedure (Table 3) [14].

Complications include mild and transient hyphema, cyclodialysis, iridodialysis, peripheral anterior synechiae, and cataract formation.

The preoperative presence of angular synechiae of more than 180° of circumference is associated with a failure rate of 100%. Some authors proposed preoperative laser treatment of synechiae with YAG laser [15].

### 2.2. Trabeculotomy

Trabeculotomy was described for the first time in 1960 by Burian; this surgical technique provided the identification of Schlemm's canal, its radial incision, and incannulation for 360 degrees with a nylon filament. Burian described an elevated success rate [16]; however, potential false passages and the difficulty to control the nylon filament made the modification of the surgical technique necessary.

In 1970 Harms and Dannheim created a scleral superior flap, similar to the flap created for trabeculectomy, so as to have a better identification of Schlemm's canal. He also introduced a new instrument: Harms' trabeculotome that acts for approximately 120° and has two parallel arms that help the surgeon by providing an external guide. If one procedure alone is not enough, it can be repeated [17].

Also Allen and Burian described trabeculotomy using a rigid probe with satisfactory results [18].

No well-designed studies to compare the efficacy of a rigid probe versus the nylon filaments have been conducted as of yet, but the small studies available in literature show a similar efficacy between the two instruments.

In 1979 Luntz reported the surgical results of standard trabeculotomy for the treatment of congenital glaucoma in 86 eyes; he described a success rate of 89.5% (IOP 18 mmHg or less under anesthesia using Schiotz tonometer). The age of the patients ranged from 2 weeks to 12 years and the mean follow-up was approximately 6.5 years [19].

Yalvac et al. reported his surgical results with standard trabeculotomy after 1, 2, and 3 years of follow-up in 24 patients the success rate was, respectively, 92%, 82%, and 74%. The end point was IOP less than 18 mmHg and more than 5 mmHg with a single intervention, stabilization of cup disc ratio, and lack of corneal enlargement [20].

A recent study by Ou and Caprioli reported a success rate ranging from 87% to 92% in case of primary congenital glaucoma presenting before one year of age [21].

In the last years a 360° trabeculotomy with an illuminated microcatheter has been described.

The use of illuminated probes allows for controlled visualization of the position of the catheter while advancing along Shlemm's canal. Dao et al. reported a 75% success rate in achieving 360° cannulation as an initial procedure in children with primary congenital glaucoma [22].

Several studies compared the efficacy of goniotomy and trabeculotomy and concluded that both are successful techniques [23, 24]. There is a general consensus to use goniotomy for initial forms with clear cornea and trabeculotomy for mild severe forms with corneal opacity.

Complications include transient hyphema, choroidal detachments or hemorrhage, and false passage into the eye; less common complications are iridodialysis and rupture of the Descemet membrane [25, 26].

### 2.3. Trabeculectomy

Trabeculectomy is a filtering procedure that is generally utilized if angle surgery in primary congenital glaucoma fails to work; however, some surgeons prefer to perform it as primary choice in aphakic glaucoma [25].

Although several studies report acceptable results, the success rate is lower than that reported in adult patients and varies from 35 to 50% [26–30]. Several studies report the enhanced success (54% to 85%) of this procedure when used as the primary intervention for congenital glaucoma [31]. Trabeculectomy presents special technical difficulties in childhood because buphthalmic eyes are bigger than usual and the lumbar anatomy is frequently impaired and it can lead to iris and ciliary body incarceration and vitreous loss [30–33]. Furthermore in childhood there is an exuberant fibrotic postoperative response with scar formation which occludes the filtering site and causes long-term trabeculectomy failure. To obviate this drawback the use of antimetabolites has been introduced. Freedman et al. retrospectively reviewed* 21 eyes of 17 patients* (mean age 2.6 years, minimum 1 month maximum 16 years) who underwent mitomycin C (MMC) trabeculectomy, selective use of postoperative 5 fluorouracile (5-FU), and diode laser suture lyses in patients suffering from refractory primary and secondary glaucoma. The follow-up period for all cases was 16.4 ± 11.4 months. The preoperative IOP of 34.1 ± 5.7 mmHg was reduced to the mean values of 16.9 ± 11.2 mmHg at last follow-up, with a mean IOP decrement of 17.2 ± 9.1 mmHg (*P* ≤ 0.001). The use of preoperative eye drops (for all cases) was reduced from 2.4 ± 0.6 before operation to 1.1 ± 1.0 after operation (*P* ≤ 0.001).

The cumulative success rate was 54.2%. A lower success rate was noted in patients younger than 1 year of age (30%) compared with those older than one year (73%) and in aphakic eyes (2%) compared with the phakic ones (64%) [34]. The reason is unknown. Beauchamp and Parks described a more exuberant healing response which together with a thicker Tenon's layer and lower scleral rigidity and thickness may be considered responsible [30]. Although others have noted poor success of MMC-augmented trabeculectomy in aphakic children, the reasons for frequent failure in these patients are unknown [35]. Susanna Jr. et al. reported an overall success rate (IOP between 4 and 21 mmHg) in 67% of 79 eyes patients (mean age of 76 months and a mean follow-up of 17 months), with devastating complications in 3 eyes [36].

The use of antimetabolites led to the improvement of the prognosis, but at the same time other complications were reported: thin avascular bleb, bleb related endophthalmitis, and long-term hypotonia and bleb leak carry substantial ocular morbidity and the potential for visual loss as well as the need for additional surgery. An increased incidence of postoperative complications is reported in mitomycin trabeculectomy comparing to trabeculectomy without antimetabolites [37–39]. Sidoti et al. reported a significant incidence of endophthalmitis in childhood compared to the rates reported in adults [28].

In the early postoperative period, the most common complications faced by the glaucoma surgeons involve either elevated IOP or hypotonia. Other complications are wound leak, choroidal hemorrhage, malignant glaucoma, cystoid macular edema, encapsulated bleb iris prolapsed, and synechiae [28–40].

Major intraoperative complications in particular expulsive choroidal hemorrhage and intraoperative choroidal effusion are more frequent in eyes with glaucoma secondary to Sturge-Weber syndrome.

The reason is due to vascular anomalies and increased pressure in episcleral veins, ciliary body veins, and choroidal veins that quickly loose fluid from the intravascular to the extravascular space when eyes are opened and intraocular pressure suddenly declines. To prevent this rare but potential catastrophic event the authors have proposed prophylactic intervention such as posterior sclerotomy, prophylactic radiotherapy or laser photocoagulation of the choroidal hemangioma, or electrocautery of the anterior episcleral vascular anomaly, also the reduction of intraoperative hypotonia by a rapid closure of the scleral flap seem to be effective to reduce the risk of expulsive choroidal hemorrhage and intraoperative choroidal effusion [41].

### 2.4. Glaucoma Drainage Implants

Glaucoma drainage implants (GDIs) provide an alternative option for IOP reduction in complicated pediatric glaucomas that are refractory to angle or filtering surgery. GDIs employ a silicon tube placed in the anterior chamber to shunt aqueous humor to the subconjunctival space where it is connected to a plate positioned in the equator region. A fibrous capsule forms around this plate. The size and the material of the plates vary between the different devices.

The first drainage system utilized was the Molteno valves in 1970 [42]. Afterwards other valves were introduced; the most utilized actually together with Molteno implants are Bearveldt and Ahmed valves [43].

The Ahmed valve is a device with a unidirectional valve restriction flow mechanism, designed to open when IOP is higher than 8 mmHg. This design is highly effective to reduce postoperative hypotonia compared to nonvalved devices which requires a two-step procedure to prevent postsurgical hypotonia and the use of medication to control IOP until the tube opens. Success rate in the different studies varies considerably from 31.3% to 92.7%; this huge difference is due to the different populations enrolled, different devices utilized, and different follow-up lengths (Tables 4 and 5) [4–47]. For instance Al-Mobarak and Khan reported a low success rate of 31% after two years in patients younger than 2 years while Al-Mobarak and Khan reported a success rate of 86% in patients with a median age of 6 years [48]. Yang and Park reported in 38 eyes with congenital glaucoma and 41 with aphakic glaucoma success rates of 92 and 90%, respectively, at 1 year of follow-up which decreased to 42 and 55% after 10 years [49]. Several studies performed on young patients did not show significant differences in postoperative IOP values [50, 51].

A meta-analysis of aqueous shunts by Minckler et al. revealed no advantages to the adjunctive use of antifibrotic agents or systemic corticosteroids [52]. The paucity of evidence that MMC improves outcomes and its potential complications have led to their more limited use [53, 54].

Freedman et al. comparison of GDIs and MMC trabeculectomy shows a major success rate of the former one in both short and long term (87% versus 36% at one year and 53% versus 19% at 6 six years) [55]. These results are confirmed in other studies. Pakravan et al. reported a success rate of 87% (IOP between 5 and 21 mmHg) in aphakic glaucoma treated with Ahmed implants versus 67% in those treated with MMC trabeculectomy 40%. He also reported an increase of complication rate in the MMC trabeculectomy group (40% versus 26.7%) [56].

The complications associated with GDIs are largely reported and seem to be more frequent in childhood compared to adulthood. The most frequent complications are shallows and flats in the anterior chamber, hypotonia, hyphema, choroidal effusion, corneal tube contact, iris abnormalities, and endophthalmitis associated with tube extrusion. Strabismus has been described after GDIs and it is due to the placement of the implant in the vicinity of the rectus muscle insertion [57–61].

In Sturge-Weber syndrome higher rate of expulsive choroidal hemorrhage, choroidal effusion, and prolonged flat anterior chamber are described. Hamush et al. reported choroidal detachment in 3 eyes of 11 patients [62]. Amini et al. reported 3 cases of choroidal detachment in 9 patients with Sturge-Weber related glaucoma who underwent Ahmed valve implantation [63]. Budenz et al. reported a serous choroidal detachment in two patients of 9 patients (20%) which underwent Baerveldt valve implant resolved spontaneously without the need to drain, the self-limiting nature of this complacence was due to prophylactic posterior sclerotomies performed, in more than one quadrant [64].

### 2.5. Deep Sclerectomy

Deep sclerectomy (NPDS) involves the unroofing of Schlemm's canal under a scleral flap, with concurrent removal of juxtacanalicular trabecular tissues and creation of a trabeculodescemetic window that provides the resistance to aqueous drainage, in order to prevent hypotonia. This procedure is technically more demanding so its use is not generalized and it is even more limited in childhood. Only few studies are reported in literature [65, 66]. A prospective study conducted in Saudi Arabia by Al-Obeidan et al. regarding NPDS as first surgical choice in 120 patients with PCG reported a success rate of 82.4% [67].

NPDS is particularly suitable in complicated glaucoma such as Sturge-Weber syndrome where hypotonia and choroidal effusion can have catastrophic consequences. Audren et al. did not report any cases of choroidal effusion of NPDS in 12 eyes of nine patients (follow-up 26 months) with glaucoma related to Sturge-Weber syndrome. So it may be considered theoretically safer than trabeculectomy and GDI and could be regarded as an alternative when possible [68].

## 3. Conclusions

Management of congenital glaucoma is still a challenge for physicians, starting from diagnosis passing through the timing and choice of the most appropriate surgical approach and ending with the long-term follow-up. Today diagnosis is facilitated with ultrasound biomicroscopy and optical coherence tomography of the anterior segment which are imaging techniques which can show the angle and surrounding structures with great detail [69, 70]. Intraocular pressure generally is measured under anesthesia; however, most anesthetic drugs lower it. Generally ketamine is avoided since it raises the values of intraocular pressure. Various instruments can be used to measure intraocular pressure in children like the rebound tonometer, the pneumotonometer, and Perkins applanation tonometer. In particular the I-care tonometer has shown to be promising in measuring IOP in awake young children [71]. Its validity and limits are well known in adult patients [72]. New surgical techniques and improvements of the traditional ones are available to manage pediatric glaucoma, which, however, remains still a challenging and niche type of surgery, probably also due to its low worldwide incidence. The different clinical situations should always be weighed against the risks associated with the procedures for the individual patients.

It is generally accepted that angle surgery remains the first choice in mild cases and both goniotomy and trabeculotomy have good success rates.

Trabeculectomy with or without MMC is preferred in refractory cases, in aphakic eyes and in older children. GDIs have a good success rate in aphakic eyes.

NPDS is still rarely used to date for long-term follow-up are available but medium term results of on-going studies are encouraging. There is also a paucity of information on sight-threatening complications. De Silva et al. evaluate the risk of glaucomatous progression in 19 patients (mean follow up of 33 years) evaluating at each control: elevation of the disk, IOP, progression of optic disk cupping, and visual fields.

Goniotomy was the first surgical approach in 27 eyes, 2 of these eyes needed a second goniotomy. Nine eyes (30%) were treated with trabeculectomy: 2 eyes with MMC 1 eye with *β*-irradiation, 1 eye secondary trabeculectomy with MMC after 19 years, and 2 eyes requiring transscleral cyclodiode laser. A total of 9 eyes (30%) showed progressive PCG, with a reduction of visual acuity >0.2logMAR units and/or progression of optic disk cupping >0.2 cup/disk ratio as a consequence of elevated IOP (>21 mmHg). The authors have found that the glaucomatous progression can occur many years after its stabilization and at any time during the follow-up period.

The authors hypothesized that the increased visual impairment with long-term follow-up is partly a consequence of sight threatening PCG progression or ocular-comorbidity that can occur at any point in the follow-up period [73].

These results underscore the importance of a life-long assessment and necessity of monitoring the progression of damage. Standard achromatic perimetry is currently the gold standard for detecting visual field loss in glaucoma and to monitoring disease progression over time. Despite advances in imaging of the optic nerve and the retinal nerve fiber layer none of the available methods has been proven to be helpful in the clinical setting for longitudinal assessment of glaucoma [74, 75].

Considerable progress has been made in the in the diagnosis and management of congenital glaucoma but potentially it remains cause of blindness, for this reason innovative studies are required to improve the existing medical and surgical options and to experiment newer.

## Figures and Tables

**Table 1:** Summary of angle surgery results in patients with primary congenital glaucoma.

Years	Author	Surgical technique	Eyes	Follow-up (years)	End point	Success rate
1953	Barkan	Goniotomy	196	17 yrs	IOP <20 mmHg	80%

1982	Shaffer	Goniotomy	287	15 yrs	IOP <20 mmHg	76.7%

1979	Lunz	Trabeculotomy	86	6.5 yrs	IOP <18 mmHg	89.5%

2007	Yalvac	Trabeculotomy	24	3 yrs	IOP <18 mmHg	92% 1 yr 82% 2 yrs 74% 3 yrs

**Table 2:** Summary of trabeculectomy surgery in primary congenital glaucoma.

Years	Author	Surgical technique	Eyes	Follow-up	End point	Success rate %
2004	Rodrigues	Trabeculectomy: 30 eyes with MMC^*∗*^ 61 eyes without MMC	91	Patients with MMC 70.2 ± 58.2 months Patients without MMC 43.8 ± 31.3 months	IOP between 15 and 21 mmHg	*∗∗*

2010	Madhy	Trabeculectomy: 15 eyes MMC and amniotic membrane transplantation 15 eyes trabeculectomy MMC^*∗*^	30	18 months	IOP between 15 and 21 mmHg	80 60

Intraocular pressure (IOP), mitomycin C (MMC), and millimeters of mercury (mmHg).

^*∗*^MMC 0.4 mg/mL for 3 minutes.

^*∗∗*^The authors did not report values of success rate; they reported *P* values obtained by Fisher exact test for categorical variables and survival analysis to access the success rate through time. No significant difference on the failure time of the procedure, for both success IOP values considered, was observed between the groups (*P* = 0.746 for IOP <21 mmHg and *P* = 0.216 for IOP ≤15 mmHg).

**Table 3:** Summary of trabeculectomy surgery in primary congenital glaucoma and secondary glaucoma including: aphakia, aniridia, juvenile open angle glaucoma, uveitis, and Sturge-Weber syndrome.

Years	Author	Surgical technique	Eyes	Follow-up	End point	Success rate %
1999	Freedman	Mmc trabeculectomy postoperative 5 FU or suture lysis	21	23 months	4< IOP >16 mmHg	52.4

2000	Snir	Trabeculectomy 5 FU or MMC plus postoperative 5 FU	12	25.8 ± 12.2 months	IOP <20 mmHg	58.3

2008	Giampani	MMC^*∗*^ trabeculectomy	114	61.2 ± 26.1 months	5< IOP <21 mmHg	55.26

Intraocular pressure (IOP), millimeters of mercury (mmHg), years (yrs), mitomycin C (MMC), and 5 fluorouracile (5-FU).

^*∗*^MMC 0.4 mg/mL for 3 minutes.

**Table 4:** Summary of GDIs implants surgery in patients with primary congenital glaucoma.

Years	Author	Type of valve implanted	Eyes	Follow-up	End point	Success rate %
2004	Al Torbak	Ahmed with corneal transplant	20	30.9 months	IOP between 5 and 21 mmHg without medical or surgery additional intervention	44 at 2 yrs 33 at 4 yrs

2014	Audrey	Bearveldt	45	30 months	IOP <21 mmHg	93.3 at 3–9 months 86.7 at 12–18 months 86.7 at 24–30 months

2014	Reza Razeghinejad	Ahmed	33	32 ± 18.3 months	IOP <21 mmHg	97 1 yr 85 2 yrs 56 5 yrs

Intraocular pressure (IOP), years (yrs), and millimeters of mercury (mmHg).

**Table 5:** Summary of GDIs implants surgery in patients with primary congenital glaucoma and secondary glaucoma including: aniridia, peter's anomaly, neovascular glaucoma, aphakic glaucoma following congenital cataract extraction, microphthalmia glaucoma after trauma, glaucoma following retinal detachment surgery, and juvenile glaucoma.

Years	Author	Type of valve implanted	Eyes	Follow-up	End point	Success rate %
1997	Eid	Molteno single or double plaits, Soker, Beraveldt	18	47.3 ± 25.1 months	6< IOP <21 mmHg	44.4

2007	Autrata	Molteno or Bearveldt	76	7.1 ± 6.5 yrs	7< IOP <21 mmHg	91 at 1 yr 82 at 2 yrs 76 at 3 yrs 71 at 4 yrs 67 at 5 yrs

2008	O'malley	Ahmed, Bearveldt, Molteno	79	5.5 yrs (mean)	IOP <21 mmHg	92–90 at 1 yrs 42–55 after 10 yrs

2009	Al Mobarak	Ahmed	42	11.1 ± 5.5 months	IOP <22 mmHg	73.8 at 1 yr 63.3 at 2 yrs

2009	Khan	Ahmed	31	11.8 ± 5.6 months	IOP <22 mmHg	90.9 at 2 yrs 58.4 at 2 yrs

Intraocular pressure (IOP), years (yrs), and millimeters of mercury (mmHg).
